RETRACTED

# Analysis of Bioelectrical Impedance Spectrum for Elbow Stiffness Based on Hilbert–Huang Transform

**DOI:** 10.1155/2022/5764574

**Published:** 2022-04-08

**Authors:** Guodong Gao, Ping Zhang, Bin Xu, Xiaogang Zhang, QuanZeng Yang, Rong Wang, ShuHuan Han, Zhen Quan

**Affiliations:** ^1^Department of Spinal Surgery, Affiliated Hospital of Gansu University of Chinese Medicine, Lanzhou, Gansu 730000, China; ^2^College of Electrical and Information Engineering, Lanzhou University of Technology, Lanzhou, Gansu 730050, China

## Abstract

With the advent of posttraumatic elbow rehabilitation, prevention of elbow stiffness has become a key part of the development of sports medicine. In order to clarify the time point of joint movement after internal fixation to the elbow and to provide a mechanical model for individualized diagnosis. This paper uses electromagnetic wave detection technology to quickly detect the bioelectrical impedance signal of the patient's lesion location, then passes the message to the upper control system for processing, summarizes the improved Hilbert–Huang transform to deep learning, and deep learning algorithms and computer technology are used to mine the bioelectrical impedance signal of the elbow joint. The simulation and human experiment results show that bioelectrical impedance signals can clarify the pathogenesis of elbow joint stiffness and the relationship between rehabilitation treatment time and duration. It has the advantages of low cost, high fitting accuracy, strong robustness, and noninvasiveness.

## 1. Introduction

Posttraumatic elbow stiffness is a posttraumatic complication of the elbow joint with high morbidity, strong disability, and concurrent functional limitations of the hand and wrist. Elbow stiffness seriously endangers human health. The data show that 15 percent of elbow dislocations patient maybe appear elbow stiffness, 21 percent of dislocations with radial head fractures maybe appear elbow stiffness, and 25 percent of humerus fractures maybe appear elbow stiffness. When the elbow joint loses its normal function, the motor function of the hand can be limited by up to 70%, and the ability of daily activities can be limited by 80% [1]. Therefore, improving the therapeutic effect of posttraumatic elbow stiffness is crucial for improving prognosis. Currently, there is no effective treatment for posttraumatic elbow stiffness. Nonsurgical and surgical methods are usually used in the clinical treatment of elbow stiffness. Nonsurgical treatment is often used for patients with loss of daily living ability of the elbow within 6 months after injury [2]. However, due to individual differences in patients and unclear signs, problems such as bleeding, rebound edema, aggravation of heterotopic ossification, and even iatrogenic fractures may occur in clinical practice. When the nonsurgical treatment effect is less effective, the surgical treatment method is used on the patient. The surgical plan is determined according to the elbow joint function score and imaging examination results. However, due to the large wounds, this method can cause extensive damage to ligaments and muscles, and even lead to ulnar nerve damage [3]. At the same time, the use of frontal and lateral X-rays and CT has increased the economic burden of patients. Therefore, when to perform joint movement after internal fixation of the elbow joint is the key point to prevent elbow joint stiffness and improve the treatment effect of elbow joint trauma.

RETRACTED

The elbow joint has a highly consistent articular surface. Three joints are wrapped in a synovial joint capsule, and there is a close relationship between the joints and the joint capsule. The ligaments of the joint are closely related to the muscles around the joint. The proximal radioulnar joint is closely surrounded by the collateral ligament complex, and the relatively narrow joint space makes the joint capsule and the ligament muscles tightly combined, which plays a secondary stabilization role [4]. After an elbow injury, hemorrhage and inflammatory mediators are involved in the repair process. Bone morphogenetic protein rises due to posttraumatic inflammatory response. Then, there are some problems: scar appearance, joint capsule contracture, heterotopic ossification, and even bioelectrical impedance change. Studies have shown that peripheral nerve injury induces fibrosis and heterotopic ossification and that delayed surgery and prolonged postoperative immobilization increase the risk of heterotopic ossification [5]. A marked increase in myofibroblasts can also trigger joint capsule stiffness. Activated mast cells are found in stiff joint capsules, which activate myofibroblasts to alter the balance of the matrix metalloproteinase system and collagen synthesis, causing collagen hyperplasia and fibrosis. The number of myofibroblasts began to increase in the early stage of injury, but the number of myofibroblasts in the stiff joint capsule did not increase in the later period [6].

With the development of cross-research between medicine and control theory, elbow joint bioelectrical impedance analysis becomes very important in clinical medicine. It can objectively describe the treatment process and analyze the weights of various factors in the treatment process [7, 8]. Since Thomasset proposed the application of the bioelectrical impedance method to the analysis of body composition in 1962, the analysis of body composition by the bioelectrical impedance method has been favored by researchers [9, 10]. The paper [11] analyzes the relationship between the bioelectrical impedance mechanism of human acupoints and anatomical histology, then provides a theoretical basis and technical support for patients with meridian imbalance and visceral lesions. The paper [12] introduces the principle of bioelectrical impedance technology in skin condition detection and describes the research and application status of this technology in skin wound detection. The paper [13] compares different bioelectrical impedance analysis parameters that demonstrate FO and their association with 30-day mortality in critical patients admitted to the emergency department. Bioelectrical impedance spectroscopy (BIS) is a technology that is widely used for the assessment of body composition. The method is based on the measurement of the electrical resistance of the body or a body region that can be quantitatively related to the amount of water in the tissues [14, 15]. The paper [16] traces the evolution of the BIS technique since its inception and presents the current state of the art, with particular emphasis on utility in clinical practice. Therefore, the physiological and pathological characteristics of patients with elbow stiffness can be characterized by bioelectrical impedance.

RETRACTED

The rest of this paper is organized as follows.  Section 2 discusses the bioelectrical impedance and its mechanism model, followed by the human body signal analysis of the elbow joint. In Section 3, a simulation experiment of the patient's elbow is discussed. In Section 4, section 5 concludes the paper with a summary and future research directions.

## 2. Bioelectrical Impedance Spectrum

### 2.1. Bioelectrical Impedance Detection

According to the source of electrical signals, the electrical properties of biological tissues can be divided into active and passive. Active response means that the current of biological tissue is generated by ions inside cells. Passive response means that the current of biological tissue is generated by external electrical stimulation (such as a current or voltage generator). Bioelectrical impedance analysis is a low-cost, noninvasive technique used to measure body composition and assess clinical conditions. It is a new diagnosis and treatment method that uses the electrical conductivity of biological intracellular fluid and extracellular fluid to detect changes in human tissue or organ function. The theoretical basis of bioelectrical impedance is that a large number of intracellular fluids and extracellular fluids contained in the human body have electrical conductivity. Under the excitation of alternating current, complex electrical impedances will be generated in biological tissues. Bioelectrical impedance analysis can reflect more inside information and express pathological states of patients. A bioelectrical impedance measurement system is shown in Figure 1.

RETRACTED

Bioelectrical impedance is a complex number consisting of resistance value *R* and reactance value *X*_*C*_. *R* is mainly caused by the total amount of water in the human body, and the *X*_*C*_ is mainly caused by the capacitance generated by the cell membrane. A simplified model of the bioelectrical impedance and its measuring instrument is shown in Figure 1. In which the membrane capacitance, intracellular fluid resistance, and extracellular fluid resistance pass through the series-parallel equivalent electrochemical model. The model has a simple structure and is easy to identify parameters.

### 2.2. Model of Bioelectrical Impedance

A single cell in each tissue of the elbow joint can be equivalent, as shown in Figure 2. In which, *R*_*m*_ represents the equivalent resistance, and *C*_*m*_ is the capacitance of the cell membrane. *R*_*i*_ represents the equivalent resistance, and *C*_*i*_ is the capacitance of the intracellular fluid. *R*_*e*_ represents the equivalent resistance, and *C*_*e*_ is the capacitance of the capacitance of extracellular fluid. The electrical signal can pass through the cell through the cell membrane and then through the intracellular fluid, or it can bypass the cell directly through the extracellular fluid. *R*_*m*_ approaches infinity at low-frequency signals, and *C*_*i*_ and *C*_*e*_ are equivalent to an open circuit in practice. Therefore, Figure 2 can be simplified to the circuit of Figure 3, which is called the three-element circuit equivalent model [17, 18].

The expression for the equivalent model of the three-element circuit is simplified as follows:

(1) $$\begin{array}{c} Z=\frac{R_{e}\left(1+jwC_{m}R_{i}\right)}{1+jwC_{m}\left(R_{e}+R_{i}\right)}\\ =\frac{R_{e}+w^{2}C_{m}R_{e}R_{i}\left(R_{e}+R_{i}\right)}{1+{\left(R_{e}+R_{i}\right)}^{2}w^{2}C_{m}^{2}}-j\frac{wC_{m}R_{e}^{2}}{1+{\left(R_{e}+R_{i}\right)}^{2}w^{2}C_{m}^{2}},\\ \left|Z\right|=\sqrt{\frac{R_{e}^{2}\left(1+w^{2}C_{m}^{2}R_{i}^{2}\right)}{1+w^{2}C_{m}^{2}{\left(R_{e}+R_{i}\right)}^{2}}},\\ \theta =-\text{arctg}\left(\frac{wC_{m}R_{e}^{2}/1+{\left(R_{e}+R_{i}\right)}^{2}w^{2}C_{m}^{2}}{R_{e}+w^{2}C_{m}^{2}R_{e}R_{i}\left(R_{e}+R_{i}\right)/1+{\left(R_{e}+R_{i}\right)}^{2}w^{2}C_{m}^{2}}\right). \end{array}$$

### 2.3. Cole-Cole Model

Through the detection of bioelectrical impedance, the recovery of the elbow joint is regularly monitored. When measuring real biological tissue, the imaginary and true parts of biology are not semicircular with frequency. It is the arc in the fourth quadrant, and the center of the circle is in the first quadrant, which is called the bioimpedance spectrogram. In this paper, the Cole-Cole bioimpedance characteristic equation is used to describe the biological tissue shown in Figure 4. As shown in Figure 4, we can see that the abscissa and ordinate of the bioimpedance is at *R*_0_ when the frequency is zero. When the frequency is infinite, the abscissa and ordinate of bioimpedance are at *R*_*∞*_.

(2) $$\begin{array}{c} Z=R_{\infty }+\frac{R_{0}-R_{\infty }}{1+{\left(jw\tau \right)}^{\alpha }}. \end{array}$$

In which, *τ*=(*R*_*i*_+*R*_*e*_)*C*_*m*_, *R*_0_=*R*_*e*_, *R*_*∞*_=*R*_*i*_*R*_*e*_/*R*_*i*_+*R*_*e*_. Eigenfrequency *f*_*c*_ is the frequency point when the imaginary part of the bioimpedance is maximum.

(3) $$\begin{array}{c} f_{c}=\frac{1}{2\pi \tau }\\ =\frac{1}{2\pi \left(R_{e}+R_{i}\right)C_{m}}. \end{array}$$

Let (3) into (2) to get (4)as follows:

(4) $$\begin{array}{c} Z=R_{\infty }+\frac{R_{0}-R_{\infty }}{1+{\left(jf/f_{c}\right)}^{\alpha }}. \end{array}$$

The trajectory of the Cole-Cole impedance circle of the biological tissue spectrum is almost in the first quadrant, so (4) can be equivalent to the result of multiple *R*_*i*_ and *C*_*m*_. Therefore, the equivalent impedance model of biological tissues is shown in Figure 5.

RETRACTED

## 3. Human Body Signal Analysis of Elbow Joint

### 3.1. Hilbert–Huang Transform

There are some methods in the field of signal processing: Fourier transform, wavelet transform, S transform, empirical mode decomposition, and variational mode decomposition. The Fourier transform is currently the most widely used signal processing method. The frequency information and phase information of the signal can be obtained from the Fourier transform. However, the Fourier transform cannot handle nonstationary signals. Nonstationary signals refer to the signal components and the frequency of each component change with time, and the Fourier transform can only receive frequency components in the entire signal segment without knowing the exact time when each component appears.

The empirical mode decomposition (EMD) method was proposed by Norden E. Huang in 1998, and the Hilbert spectrum was introduced into the EMD method to form today's Hilbert–Huang transform (HHT). HHT methods include empirical mode decomposition (EMD) and the Hilbert transform (HT). The HHT method is an adaptive signal processing method. It has obvious time-frequency characteristics after the Fourier transform and the wavelet transform. EMD plays an important role in this process [19, 20].

RETRACTED

### 3.2. Hilbert–Huang Transform

In this paper, Figure 6 shows the flow chart of our proposed algorithm.

**Step 1 .**

The very large value point of the original signal *x*(*t*) obtained in turn is recorded as *x*_*t*_(1) to *x*_*t*_(*n*_1_), and the very small point of the original signal *x*(*t*) collected is obtained in turn, and the minimum point of the original signal *x*(*t*) is recorded as *x*_*b*_(1) to *x*_*b*_(*n*_2_). In which, *n*_1_ represents the number of maximum points of *x*(*t*) , and *n*_2_ represents the number of minimum points of *x*(*t*).

**Step 2 .**

Get the upper envelope of the original signal *x*(*t*) from *x*_*t*_(1) to *x*_*t*_(*n*_1_), which is recorded as *x*_1_(*t*) .The lower envelope of the original signal *x*(*t*) is obtained from *x*_*b*_(1) to *x*_*b*_(*n*_2_) , shown as *x*_2_(*t*). Then, the mean of the envelope is recorded as *m*_0_′(*t*) which is defined by (5). And repeat until |*n*_1_ − *n*_2_| ≤ 1.

(5) $$\begin{array}{c} m_{0}^{\prime }\left(t\right)=0.5\times x_{1}\left(t\right)+0.5\times x_{2}\left(t\right). \end{array}$$

**Step 3 .**

There is a scale coefficient of *k*_1_ to *k*_*n*_, and the initial value of *k*_1_ to *k*_*n*_ is 1. Then, coefficient are multiplied by all extreme points, so we can get envelope *m*_1_′(*t*). Then, we can get the norm expression in (6).

(6) $$\begin{array}{c} \nabla ={\left(\int_{0}^{t_{s}}{\left|m_{1}^{\prime }\left(t\right)-x\left(t\right)\right|}^{1/2}dt\right)}^{2}. \end{array}$$

In which, *t*_*s*_ is the final moment of sampling. *n* is the number of all extreme points, and *n*=*n*_1_+*n*_2_.

**Step 4 .**

Through the coefficient of *k*_1_ to *k*_*n*_, get the relational expressions of ∇(*k*_1_, *k*_2_, *k*_3_,…, *k*_*n*_). ∇ can be minimized by adjusting the proportional coefficient of *m*_1_′(*t*) based on Newton iteration method in (7).

(7) $$\begin{array}{c} k_{1_{m+1}}=k_{1_{m}}-\frac{\nabla {\left(k_{1}\right)}_{m}}{\nabla^{\prime }{\left(k_{1}\right)}_{m}}\\ k_{2_{m+1}}=k_{2_{m}}-\frac{\nabla {\left(k_{2}\right)}_{m}}{\nabla^{\prime }{\left(k_{2}\right)}_{m}}\\ k_{3_{m+1}}=k_{3_{m}}-\frac{\nabla {\left(k_{3}\right)}_{m}}{\nabla^{\prime }{\left(k_{3}\right)}_{m}}\\ \vdots \\ k_{n_{m+1}}=k_{n_{m}}-\frac{\nabla {\left(k_{n}\right)}_{m}}{\nabla^{\prime }{\left(k_{n}\right)}_{m}}. \end{array}$$

In which, $k_{i}\in \left(\begin{array}{cc} 0.2 & 10 \end{array}\right)$ is the final moment of sampling. *m* is the number of current iterations.

**Step 5 .**

Get the envelope of *m*_1_(*t*) based on *x*_*t*_(*n*_1_), *x*_*b*_(*n*_2_) and coefficient of *k*_1_ to *k*_*n*_ .Then, calculate the difference between *m*_1_(*t*) and *x*(*t*) as *m*(*t*) . Similarly, calculate *m*_2_(*t*) to *m*_*Z*_(*t*). *Z* is the number of the IMF.

RETRACTED

**Step 6 .**

The Hilbert transformation is combined from *m*_1_(*t*) to *m*_*Z*_(*t*), and the result as (8).

(8) $$\begin{array}{c} E\left(t,w\right)=\sum_{i=1}^{Z}\text{hilbert}\left(m_{i}\left(t\right)\right). \end{array}$$

### 3.3. Experimental Simulation

Figure 7 shows the effect graph from generation to stop of a single excitation signal under normal circumstances. The coordinate system *x* axis represents the signal *t* axis, the coordinate system *y* axis represents the signal *w* axis, and the coordinate system *z* axis represents the amplitude of the signal. As shown in Figure 7, the excitation signal operates steadily in the model at a frequency of 40 Hz. When the excitation signal stops instantaneously, no abnormal signal is generated.

Figure 8 shows abnormal information generation time under improved HHT. As shown in Figure 8, the coordinate system *x* axis represents the signal *t* axis, the coordinate system *y* axis represents the signal *w* axis, and the coordinate system *z* axis represents the amplitude of the signal. As shown in Figure 8, abnormal signals change over time, making it easy to get the abnormal signal generation moment.

Figure 9 shows W axis projection under improved HHT. As shown in Figure 9, the coordinate system *x* axis represents the signal *t* axis, the coordinate system *y* axis represents the signal *w* axis, and the coordinate system *z* axis represents the amplitude of the signal.  Table 1 shows abnormal signal *w* axis projection amplitude frequency. As shown in Figure 9 and Table 1, the distribution of abnormal signals on the *w* axis, and the similar signals can be subdivided. Therefore, it is easier to analyze the cause of abnormal signals.

Figure 10 shows abnormal information under improved HHT. As shown in Figure 10, the coordinate system *x* axis represents the signal *t* axis, the coordinate system *y* axis represents the signal *w* axis, and the coordinate system *z* axis represents the amplitude of the signal.  Table 1 shows abnormal signal *w* axis projection amplitude frequency. As shown in Figure 10 and Table 2, the spectral results by the improved HHT are much lower than the traditional HHT results, and the swing error after signal processing is greatly weakened.

## 4. Experiments

The bioelectrical impedance spectrum (BIS) analysis system of the elbow joint is shown in Figure 11. The electrical conductivity of tissues with different dielectric properties is significantly different. Therefore, a bioelectrical impedance acquisition system for patients with elbow stiffness is built, and excitation electrodes are applied on the surface of the patient's elbow. The voltage signal, the corresponding electrical impedance, is calculated, and the HHT is used for analysis in the frequency domain, and finally the required physiological and pathological characteristics of the elbow joint are obtained.

RETRACTED

Most of the traditional BIS measurement methods are based on time-division and single-frequency technology. The excitation signal generated each time has only one frequency, and the impedance measurement is completed by changing the frequency continuously many times. The measurement frequency is changed, so the measurement speed is relatively low. When switching measurements at different frequency points, it takes a long time to establish new electrical impedance information, but the state of tissues and organs of the organism changes dynamically, and the impedance information of the organism is captured in time. Therefore, it is impossible to accurately measure the electrical impedance information of an organism at a specific time. With the development of bioelectrical impedance technology research, two or more frequency signals are used as excitation sources to extract bioelectrical impedance information. A multifrequency BIS measurement system is proposed to realize the measurement of BIS.

### 4.1. Excitation Signal Source

Due to the characteristics of human body characteristics, the signal has the following characteristics: with the characteristics of near-field detection, the signal is basically undetectable when it is far away from the surface of the human body. The human body signal is usually weak, at most mV level. It is a low-frequency signal, and the energy is mainly a few Hz below 100 Hz. The interference signal overlaps with the signal of the human body, and the interference is particularly strong. The interference comes from inside the organism, such as electromyography interference and breathing interference.

In this paper, the signal source is the multisine signal, and its time-domain spectrogram is shown in Figure 12, and its frequency-domain spectrogram is shown in Figure 13. Multisine signals are formed by mixing multiple equal-amplitude sinusoidal signals of different frequencies and phases. Among them, the frequency of each sine signal is twice the frequency of the previous sine signal, which provides feasibility for whole-cycle sampling. In Figure 12, the horizontal axis is the sampling point. The vertical axis is the amplitude.

In Figure 13, the horizontal axis is the frequency. The vertical axis is the amplitude.

### 4.2. Hardware Acquisition Circuit

An experimental principle flow chart is shown in Figure 14. The FPGA converts the predesigned multisine excitation signal into an analog signal through the DAC module and then through the operational amplifier. Next, the processed signal is injected into the elbow joint through the human body metal clip. The processing platform converts the collected signal to the ADC module and then transmits it to the FPGA or PC platform for signal analysis.

RETRACTED

A schematic diagram of constant current source is shown in Figure 15. The transmission of the excitation signal and the reception of the target signal are realized through the above circuit.

### 4.3. Data Collection

A bioelectrical impedance spectrum analysis system is used to get experiment results by volunteer. In the future, the sample will be extended to people of different ages, occupations, physical conditions, and genders, increasing the experimental samples and improving the versatility of the experiment. The experiment procedure is shown in Figure 16.

The constant current source, OSC, FLASH, voltage conversion module, SPARTAN-6, and RS485 interface circuit diagram jointly realize the emission of an excitation signal and the reception of a target signal. The acquisition system hardware PCB is shown in Figure 17.

Physical map of signal generating device is shown in Figure 18.

Observing the input and output waveforms through the oscilloscope RIGOL DS1102 E, the waveform of the oscilloscope waveform is shown in Figure 19.

### 4.4. Data Collection

A comparison of receiving and sending signals with ordinary resistance is shown in Figure 20. The red signal represents the waveform of the excitation source signal, and the blue signal represents the waveform of the received signal.

A comparison of receiving and sending signals with the human body is shown in Figure 21. The red signal represents the waveform of the excitation source signal, and the blue signal represents the waveform of the received signal. This system can clearly obtain the impedance characteristics of the human body.

## 5. Conclusion

With the development of artificial intelligence, more and more technologies are being applied to the health field. Driven by artificial intelligence technology, the collection and analysis of clinical information has achieved qualitative improvements. Using artificial intelligence for data analysis can more effectively detect and classify lesions, and then make a more accurate quantitative analysis of the disease. Accurate assessment of the treatment effect can be made earlier by making more accurate diagnoses and predictions of patients. In clinical trials, these techniques can help to evaluate the effects of treatments in less time and with fewer patients, reducing the cost of clinical trials. Posttraumatic elbow stiffness is a posttraumatic complication of the elbow. Under normal circumstances, the soft tissue around the elbow joint mainly bears tensile stress. If the joint is fixed for a long time in the shortened position of the tissue, the tensile stress acting on the tissue will be eliminated, the tissue will contract, and eventually elbow joint stiffness will appear. Estimation is the key to predicting such diseases. By applying noninvasive and controllable and periodic tensile stress to the periarticular tissue, the remodeling of the periarticular tissue is a key mechanism in the treatment of this type of disease.

RETRACTED

In this paper, electromagnetic wave detection technology is used to quickly detect the bioelectrical impedance signal of the patient's lesion location, and deep learning algorithms and computer technology are used to mine the bioelectrical impedance signal of the elbow joint. From the perspective of bioelectrical impedance, all this can clarify the pathogenesis of elbow joint stiffness and the relationship between rehabilitation treatment time and duration. In summary, the bioelectrical impedance spectrum can perform early disease diagnosis, biological tissue fluid monitoring, and physiological state assessment through patient signals. It has the advantages of low cost, high fitting accuracy, strong robustness, and noninvasiveness.

## Figures and Tables

**Figure 1:** Bioelectrical impedance measurement system.

**Figure 2:** Parallel equivalent impedance circuit.

**Figure 3:** Three-element circuit equivalent model.

**Figure 4:** Complex impedance trajectory of biological tissue.

**Figure 5:** Equivalent impedance model of biological tissues.

**Figure 6:** Flow chart of our proposed algorithm.

**Figure 7:** Status signal.

**Figure 8:** Abnormal information generation time under improved HHT.

**Figure 9:** W axis projection under improved HHT.

**Figure 10:** Abnormal information under improved HHT.

**Figure 11:** Elbow joint bioelectrical impedance spectrum monitoring system.

**Figure 12:** Multisine time-domain signal.

**Figure 13:** Multisine frequency domain signal.

**Figure 14:** Experimental principle flow chart.

**Figure 15:** Schematic diagram of constant current source.

**Figure 16:** Human body measurement.

**Figure 17:** Acquisition system hardware PCB diagram.

**Figure 18:** Physical map of signal generating device.

**Figure 19:** Oscilloscope waveform.

**Figure 20:** Oscilloscope waveform.

**Figure 21:** Oscilloscope waveform.

**Table 1:** Abnormal signal *w* axis projection amplitude frequency.

Frequency	50	65	160	174	180	300	325
Amplitude	380	655	210	586	425	565	403

RETRACTED

**Table 2:** Amplitude frequency under improved HHT (*w*=100).

Time	40	45	50	55	60	65	70
Amplitude	0	0	123	425	665	433	314

## Data Availability

The simulation experiment data used to support the findings of this study are available from the corresponding author upon request.
